# Machine Learning Techniques for Human Age and Gender Identification Based on Teeth X-Ray Images

**DOI:** 10.1155/2022/8302674

**Published:** 2022-01-04

**Authors:** K. C. Santosh, Nijalingappa Pradeep, Vikas Goel, Raju Ranjan, Ekta Pandey, Piyush Kumar Shukla, Stephen Jeswinde Nuagah

**Affiliations:** ^1^CS&E Department, Bapuji Institute of Engineering and Technology, Davangere, Karnataka, India; ^2^Department of Information Technology, KIET Group of Institutions, Delhi-NCR Meerut Road (NH-58), Ghaziabad 201206, Uttar Pradesh, India; ^3^School of Computing Science and Engineering, Galgotias University, Greater Noida, Uttar Pradesh, India; ^4^Applied Science Department, Bundelkhand Institute of Engineering and Technology, Jhansi, Uttar Pradesh, India; ^5^Computer Science & Engineering Department, University Institute of Technology, Rajiv Gandhi Proudyogiki Vishwavidyalaya, Technological University of Madhya Pradesh, Bhopal 462033, India; ^6^Department of Electrical Engineering, Tamale Technical University, Tamale, Ghana

## Abstract

The use of digital medical images is increasing with advanced computational power that has immensely contributed to developing more sophisticated machine learning techniques. Determination of age and gender of individuals was manually performed by forensic experts by their professional skills, which may take a few days to generate results. A fully automated system was developed that identifies the gender of humans and age based on digital images of teeth. Since teeth are a strong and unique part of the human body that exhibits least subject to risk in natural structure and remains unchanged for a longer duration, the process of identification of gender- and age-related information from human beings is systematically carried out by analyzing OPG (orthopantomogram) images. A total of 1142 digital X-ray images of teeth were obtained from dental colleges from the population of the middle-east part of Karnataka state in India. 80% of the digital images were considered for training purposes, and the remaining 20% of teeth images were for the testing cases. The proposed gender and age determination system finds its application widely in the forensic field to predict results quickly and accurately. The prediction system was carried out using Multiclass SVM (MSVM) classifier algorithm for age estimation and LIBSVM classifier for gender prediction, and 96% of accuracy was achieved from the system.

## 1. Introduction

Technological advancement in modern medicine helps medical professionals to diagnose the nature of the medical condition of a person more effectively and medicate accurately. Technical advancement in the field of medicine shows several types of evolution in radiologic technology, such as radiographic fluoroscopy, molecular imaging, and digital imaging. The present study was conducted by using digital radiographs of teeth, also known as orthopantomogram (OPG), considered as input for gender identification and age estimation of humans. However, the traditional method followed by forensic practitioners for identification is time-consuming; hence, a complete automated system was developed for personal identification, which produces results quickly and accurately.

The human body has a tendency to undergo changes in lifetime due to any external cause or internal metabolism changes. In such case, teeth are the only structure that will not be affected by any causes due to their hardness nature and low metabolism [1]. Dental X-ray images provide useful information in identification, and it is considered a good material in either living or nonliving populations for genetic study and odonatological, anthropological, and forensic investigation. Identification based on teeth images has higher accurate results than any other parts in humans. Teeth development stages and dental eruption factors depicted in a few atlases help manual investigation process in forensic dentistry. Identification of an individual in forensic medicine is most challenging and confidential in the matter of civil law and crime investigation [2, 3]. Hence, prediction based on observing anatomical features of teeth should be conducted with higher accuracy. Teeth images are publicly unavailable and have to be collected from the dental college, dental hospitals, or clinics that have X-ray imaging facilities.

Forensic odontology is a department in dentistry that is associated with the scientific study of the anatomy of teeth that should handle properly and analyze eruption of teeth as evidence of gender determination and age assessment. Various techniques exist in estimation of age like anthropological study, psychological and radiological method, and odonatological and skeletal analysis [4, 5]. The cuspids or eyeteeth mainly show the sexual difference from other teeth in humans. These teeth are rugged in nature and have resistance to disease. The main goal of this paper is to deliver a state of art evidence and trends and to fill gaps in the experiments on age and gender determination that was based on machine learning methods. In particular, medical image analysis is the trending and challenging research area in machine learning communities. Though the dental structures and features are almost the same in males and females, few changes in the size of the tooth will exhibit some clues about gender differences. Forensic experts manually identify gender and age differences by tooth dimensions and craniofacial morphologies [6, 7].  Figure 1 illustrates a standard numbering for each tooth. Panoramic image of teeth is divided into four quadrants; each quadrant has 8 sets of teeth. A number of denotation systems for teeth are available in the dentition field, but FDI (Federation Dentaire International) is a global standard labeling system used by many researchers. FDI uses a 2-digit global standard labeling system for tooth identification, where the first number represents the quadrant of the tooth and the second number represents the number of the tooth from the midline, as depicted in Figure 1.

A sample of FDI dental labeling on an adult panoramic image is depicted in Figure 1. It has four quadrants, upper jaw right (Q1), upper jaw left (Q2), lower jaw left (Q3), and lower jaw right (Q4). It can be evaluated in a clockwise direction [8]. The teeth number begins from 1 to 8 in each quadrant that starts from the middle line and moves towards the distal end. For example, an upper jaw right is a wisdom tooth that can be called tooth number “18” or a lower jaw left tooth that can be numbered as “38.” A complete set (32 teeth) of an adult human is depicted in Figure 2.

Human teeth have two parts, upper jaw and lower jaw, called maxillary and mandible jaw, respectively. Each jaw has 8 teeth on the left side and 8 teeth on the right part with a universal numbering and palmer numbering system [9].  Table 1 illustrates the numbering system of each tooth.

Orthopantomogram, known as OPG, and cephalogram are two different types of X-ray images in dental analysis. OPG creates a panoramic vision of teeth, which consist of both the maxillary jaw and mandible jaw, whereas a cephalogram is an X-ray image of facial structure. Age and gender determination required a complete view of teeth rather than a partial view like cephalogram [10, 11]. Hence, OPG is used widely in individual identification.  Figure 3 depicts the different types of dental X-ray imaging available.

Figure 3(a) is bitewing X-ray imaging that depicts details of lower teeth and upper teeth in a particular part of the mouth. The exposed area in bitewing X-ray imaging shows the features of teeth from the crown to the root of teeth. In Figure 3(b), periapical X-ray imaging type, one can notice minute parts inside a tooth that depicts the entire tooth with roots and soft tissues. Every periapical tooth image depicts a complete portion of a tooth, either lower jaw tooth or upper jaw tooth.  Figure 3(c) is the orthopantomogram X-ray image. This type of imaging displays a complete panoramic view of teeth [12–14]. Dataset of orthopantomogram (OPG) was used in this paper for detection of gender and age estimation.

## 2. Literature Review

Many researchers have focused on the manual method of identification using teeth, but very few contributions were made on machine learning approaches and computer vision for automated gender and age identification based on teeth. In this section, we briefly focus on the latest articles that illustrate the methodology, technical aspects, and other significant contributions of researchers in the prediction of age and gender.

Wallraff et al. [15] in 2021 proposed a method for age determination based on panoramic digital X-ray images of teeth using deep learning. The authors used a supervised regression-based deep learning technique by considering a dataset of 14000 images.

Saloni et al. [16] in 2020 proposed a method based on digital images of teeth in the identification of teeth by analyzing morphometric means of mandible ramus of 250 OPG samples. The mandible ramus may be used as an alternate tool in determining gender based on the OPG of the selected population. The authors studied mandible ramus measurements by discriminant function analysis. This outcome indicates that mandible ramus exhibits better sexual dimorphism. In 2020, Poornima Vadla et al. [17] introduced a technique based on permanent mandible teeth of the left-sided jaw. Their study focused on estimating age with high accuracy based on the Camerier method applied from an Indian-specific formula on the left and right sides of mandibular teeth. The authors used radiographs of 50 samples (25 males and 25 females) of range 5–15 years. The outcome values were recorded based on the Camerier technique in estimation of age based on Indian-specific equations. Okkesim and Erhamza [18] in 2020 conducted a study for determination of human gender based on mandibular ramus. Mandibular teeth play a vital role in determining human gender since mandible bone is the largest, dimorphic, and strongest bone in the skull. Most recent studies highlighted that CBCT (cone-beam computed tomography) is better than any traditional technique. Some of the important features in mandible teeth like-gonial angle, ramus measurement, and a few morphologic parameters are reported. Researchers studied different parameters in the mandible. Vila et al. [19] built a gender classification technique based on CNN approaches like the DASNet method and VGG-16 architecture methods. Their classification system was carried out using 3500 OPG images. Patil et al. [20] conducted a study to determine the gender of humans using discriminant analysis and logistic regression based on mandible parameters. They conducted a study using 509 panoramic images. The accuracy of their experimental results is tabulated in Table 2.

In 2020, Neves et al. [21] developed a predictive model for gender identification based on mesiodistal widths using a permanent dental cast. A total of 168 dental casts were considered for classification. Mesiodistal width of first right molar to left molar was calculated for every cast. In 2020, Dalessandri et al. [22] reviewed articles on 2D radiological method versus 3D radiological for determination of age based on teeth of 18 years old. The authors' review assesses the present trend with reliability and accuracy of OPG versus CBCT for determination of age and gender. The final outcome of their survey illustrated that CBCT was found to be accurate when compared with OPG in teeth anatomy evaluation. Stella and Thirumalai [23] developed an automation tool for estimation of age based on dental OPG images. The authors developed two methods for individual age assessment using the Demirjian and Nolla methods. This application was developed by using MS excel Visual Basic Application (VBA). This helps in the automation technique using any programming environment. Bali Behl et al. [24] proposed a method based on panoramic evaluation for mandible morphometric changes in postpubertal and prepubertal in the Turkish population. The authors measured bicondylar breadth (BB), gonial angle measurement, antegonial angle (AGA), ramus height, and ramus breadth (RHRB), which were captured from the Turkish population. They conducted this experiment on 750 digital radiographic images of ages from 5 years to 50 years. All parameters values from OPG radiographs were recorded and analyzed using the software Java Image Process. In 2019, Andrade et al. [25] developed a system for determination of gender and age estimation using pulp cavity volumes based on the CBCT method. They used 120 experimental samples of CBCT scans from the Brazilian population of both genders of ages ranging from 13 years to 70 years. Pearson's correlation evaluation methods were used in assessing the relation between pulp volume and chronological age. Higher accuracy can be achieved by using this formula when it is applied to pulp volume for one or both teeth. Good results can be fetched for samples of age more than 35 years in age estimation.

## 3. Feature Extraction

Feature extraction is the process of identifying key features in the dataset available. It is a part of the dimensionality reduction process in which an initial set of images were divided into many manageable groups. Determination of humans based on skeletal parts available is the most challenging task for forensic experts when only fragmented parts of the body are recovered [26]. In this situation, forensic dentistry will help in gender identification and age estimation based on the dental remaining and skull part. Some of the salient and dominant features in teeth for the identification process are illustrated in this section. In this paper, the most dominant features of teeth which help in determination of age and gender were identified. Few features identified from teeth are intercanine distance, incisor width, and canine width; they play a significant role in judging age and gender using teeth. Feature values extracted and recorded the values of these features in a feature matrix form. The next phase in the identification process is the conversion of feature matrix values to an understandable classifier format [27].

The odontometric features identified and analyzed for gender and age assessment are as follows:

- Incisor width: central incisors' width from both mandible and maxilla was analyzed and measured. The measurement of the incisor in the mandible differs from the maxillary jaw in males and females.
- Distance measured between canine: distance between canine from maxilla and mandible jaw is noted. This intercanine distance is the measurement between teeth numbers 13 and 23 in the maxillary jaw and the distance between teeth numbers 33 and 43 in the mandible. Figures 4(a) and 4(b) represent the samples of measurement of maxillary incisor teeth and mandible intercanine distance.

## 4. Materials and Methods

The present experimental study for the prediction of individuals was conducted based on digital X-ray images of teeth. Dental X-ray images were publicly not available. Hence, they were collected from local dental colleges and dental clinics, which have digital X-ray imaging facilities [28]. The local dataset was obtained with proper proceedings and academic agreement between two dental colleges. A total of 995 samples of teeth were collected from the College of Dental Sciences, Davangere, and 147 samples were collected from Bapuji Dental College and Hospital, Davangere, Karnataka, India. In total, we have 1142 datasets available for research analysis.

Figure 5(a) depicts the distribution of datasets based on the age of 5-year interval, segregating male and female count per group. The age distributions of available 1142 datasets of teeth were divided into 11 groups of 5 years of range per group except the first and last groups since the first group is datasets of the age group of 1–10 years and the last group is for the age group of 60 years and above.  Figure 5(b) illustrates the total samples of males and females (total 632 male and 510 female samples).

### 4.1. Methodology

The proposed system for age assessment and determination of gender has a systematic methodology depicted in Figure 6. Basic blocks in methodology are data collection, preprocessing of input image [29], features extraction, feature matrix, conversion of feature matrix into understandable classifier format, and classification. Out of 1142 local samples, 80 percent of dataset samples (913 samples) were used as the training dataset, and 20 percent of dataset samples (229 samples) were used as the unseen testing dataset. Subjects that came under the decayed tooth, missing tooth, or broken tooth were excluded from the experimental study. A normal healthy state and caries-free teeth were considered for the study. An OPG of teeth was provided as input for the model. The initial stage of the identification system was preprocessing the image. This input sample was preprocessed by removing unwanted labels and noise present in the sample. The outcome of preprocessing stage was an enhanced image, which was essential for better accuracy in prediction. The most important and dominant features in teeth that helped in the identification process were extracted. Feature values of teeth like incisor width and intercanine distance were extracted from an input OPG image. Feature matrix was constructed, and feature matrix values were converted to classifier understandable format. Figure 6 depicts the methodology for age and gender identification. Finally, the model classified age and gender from an input OPG image. The age and gender identification system were implemented using a Support Vector Machine (SVM) classifier.

Gender identification based on teeth was carried out using the LIBSVM classifier tool and training with several kernels and with different values of hyperparameters [29]. Since gender determination required two classes, the age estimation process was carried out using the Multiclass SVM (MSVM) classifier tool, and images were trained with several kernels and with different hyperparameter values. Age estimation required multiple classes. Hence, the LIBSVM classifier and MSVM classifier were used for gender and age identification [30], respectively.

Few samples of teeth datasets collected from College of Dental Sciences, Davangere, and Bapuji Dental College and Hospital, Davangere, are shown in Figures 7 and 8, respectively. These images were received in Tagged Image File Format (TIFF) format.

## 5. Experimental Results and Discussion

The human age and gender classification model is a fully automated system that predicts the gender of humans with an estimation of age. The model displays the result by taking only the input of an OPG of teeth. It produces results in less than a minute with higher accuracy. Classification techniques used and outputs obtained from classifiers with various kernels and hyperparameters are highlighted in this section. Age estimation and gender determination are carried out by MSVM and LIBSVM, respectively. The initial stage in the prediction model is to preprocess the input image by removing image noises, which may be adjoined while capturing images. The subsequent task of image preprocessing is to enhance the brightness and quality of the image [31].

### 5.1. Pixel Brightness Transformation

Brightness transformations modify pixel brightness, and the transformation depends on the properties of a pixel. Contrast enhancement is an important area in image processing. It is widely used for medical image processing. The function used is *cv*2*.cvtColor (img, cv*2*.COLOR_BGR*2*GRAY)*. The outcome of this stage is an enhanced version of the original image. The result after the preprocessed image is depicted in Figure 9.

#### 5.1.1. Edge Detection Using Canny Edge Detection Algorithm

Image segmentation is a technique of partitioning the images into multiple segments. Specifically, the image segmentation method is used to locate objects and boundaries of images. The Canny detection algorithm is used to detect edges of teeth, which aids the model in predicting age and gender accurately.

The Canny edge detection technique uses five steps for the detection of edges of input images. The following steps are used in this paper to detect edges from teeth OPG.  Figure 10 depicts the outcome of the Canny edge detection technique performed on an OPG image.

Steps in edge detection using the Canny edge detection algorithm are as follows:

1. Conversion of image based on Gaussian filter.
2. Sigma = 1.5, G Kernel size (5 × 5)
3. Gradient Calculation.
4. Horizontal filter *K*_*X*_ and Vertical filter *K*_*Y*_
5. Ix = filters.convolve (image, *Kx*).
6. Iy = filters.convolve (image, *Ky*).
7. Nonmax suppression: To achieve thin edges
8. *angle* = *A* *∗* 180*/np.pi*
9. angle [angle <0] + = 180
10. Double Threshold
11. high_Threshold = image.max( ) *∗* highThresholdratio; low_Threshold = high_Threshold *∗* hlowThresholdratio;
12. Tracking edge-based hysteresis
13. Low_*T* = Low_T *∗* max(max(*b*-*w*))
14. High_*T* = Low_T *∗* max(max(*b*-*w*))

#### 5.1.2. Mathematical Modeling for Prediction Based on Teeth

Mathematical equations involved in prediction of age and gender are described in this section. Equation (1) is used in calculation for gender differences that appeared on the left and right part of maxillary and mandible canines:

(1) $$\begin{array}{c} \text{gender difference}=\frac{\left(Xm/Xf-1\right)}{100}, \end{array}$$

where *Xm* is the average of canine teeth width in males and *Xf* is the average of canine teeth width in females.

Noise removal from digital images is done by applying a Gaussian filter, as shown in equation (2). To perform this operation, the image convolution method was used by applying a Gaussian kernel of 3 × 3, 5 × 5, 7 × 7, and so on. Sizes of Gaussian kernel depend on image blurring effects. In the present model, a 5 × 5 kernel size has been used. The formula for Gaussian kernel filter (2*k* + 1) *∗* (2*k* + 1) is given as

(2) $$\begin{array}{c} Hij=\frac{1}{2\pi \sigma }\text{exp}\left(-\;\frac{{\left(m-\left(k+1\right)\right)}^{2}+{\left(n-\left(k+1\right)\right)}^{2}}{2\sigma^{2}}\right). \end{array}$$

Some part of mathematics is involved behind the scene, mainly depending on derivatives. This mathematical-based formula was converted to equivalent python codes.  Table 3 is the comparison between feature values of central incisor width and intercanine width in millimeters.

### 5.2. SVM Training

#### 5.2.1. LIBSVM Training for Gender Determination

The LIBSVM classifier is used for gender determination from teeth images. LIBSVM is trained with different kernels of SVM, namely, Linear, Polynomial, Gaussian Radial Basis Function (RBF), and Sigmoid kernels. These are trained with different parameters of SVM like *C*, *γ*, and *d*. The LIBSVM executable *svmtrain* is employed for SVM training with various svm_type and kernel_type. Kernel parameters also have a significant effect on the decision boundary. Two features values from the teeth were extracted for age and gender determination [29]. The values of these features are extracted from the GUI from a teeth X-ray image. The training (memorization) accuracy of the SVM classification engine is calculated using the following expression:

(3) $$\begin{array}{c} \text{training accuracy}=\frac{\text{Tc}}{Ts}\;\times \;100, \end{array}$$

where *T*_*C*_ represents the total number of samples correctly classified by the SVM and *T*_*S*_ represents the total number of samples used for testing.

Figure 11 depicts the training dataset feature matrix of teeth for gender identification. Each row in the feature matrix represents the feature of each image in the dataset [30]. The first column represents the class for gender determination, where 0 is for male and 1 indicates female. The second and third columns represent the feature values extracted from teeth.

LIBSVM classifier uses two classes for gender, and the description of the class label used in the LIBSVM classifier is depicted in Table 4, since gender determination has only two classifications.

#### 5.2.2. MSVM Training for Age Estimation

The MSVM classifier is used for age estimation from teeth images. Different kernels of MSVM, namely, Linear, Polynomial, Gaussian Radial Basis Function (RBF), and Sigmoid kernels, are used for training teeth datasets. The training dataset feature matrix of teeth is depicted in Figure 12, where 832 indicates the number of data (images in the dataset) and 2 indicates the dimension (number of features) of the data. Each row in the feature matrix represents the feature of each teeth image in the dataset [31]. The last column represents the class of the age classification.

MSVM classifier uses multiple class labels for age estimation. The class label description used in the M-SVM classifier is depicted in Table 5, since age estimation has multiple age groups, and hence it is classified using multiple class label SVM.

### 5.3. SVM Testing

For the testing phase, 20 percent of unseen data samples were used for gender and age classification system.

#### 5.3.1. LIBSVM Testing for Gender

The LIBSVM executable command svm-predict.exe is used for testing and validating the classification results. Once the best hyperparameters are determined using the grid search technique, the training model with the best cross-validation accuracy [15] is considered for LIBSVM testing.

Accuracy from teeth unseen dataset is depicted in Table 6 and in Figure 13, respectively. From Table 6, we can notice that the RBF kernel shows the best classification results of accuracy of 95.83 percent for the teeth dataset. Since the classification result is above 95 percent, the models generated for the teeth dataset using RBF kernel by LIBSVM training are acceptable. Comparisons of different LIBSVM kernels for gender determination with various hyperparameters are illustrated in Figure 14. Figures 14(a)–14(d) show the accuracy of gender classification performed by using Polynomial, Linear, RBF, and Sigmoid kernels, respectively. The highest accuracy of 95.83% is achieved for gender classification from the RBF kernel for hyperparameter values *d* = 3, *c* = 28, and *g* = 0.04167.

#### 5.3.2. MSVM Testing for Age

The MSVM executable command *predmsvm.exe* is used for testing and validating the classification results. The best hyperparameters are selected using the grid search technique, and the training model with the best cross-validation accuracy is considered for MSVM testing.  Figure 15 depicts the age classification test case results validated for unseen dataset samples of teeth. MSVM classifiers with various kernels are used to build the best model for accuracy.

RBF kernel yields best classification results of accuracy of 97.91 percent for teeth testing dataset as depicted in Table 7. Since the classification result is above 97 percent, the models generated for femur and teeth dataset using RBF kernel by MSVM training can be acceptable.

## 6. Conclusion and Future Scope

From the present study, the morphological differences in identifying age and gender in the teeth were observed. Incisor width and intercanine distance in male teeth were found to be more compared to female teeth. The majority of all the parameters from the teeth of the male tended to be slightly more than female. The formula that was developed and used in this paper provided good and accurate results in prediction by using LIBSVM classifier and MSVM classifier. 95% of accuracy was achieved for gender determination, and 97% of accuracy was achieved for estimation of age. In conclusion of this paper, we were able to meet the goal of prediction by achieving the experimental results, which were nearly matching to ground truth values. This system may be used further as a novel model in personal identification without human intervention. It can be effectively used and applicable in the forensic science department for accurate and fast test results. In this paper, we have developed a system that makes the task easier in studying and analysing the femur digital radiographs for age and gender identification. This paper can be elaborated by identifying and extracting some more important teeth features and by standardizing those new features from the datasets. Furthermore, this research work can be elaborated on other parts of the human body, such as pelvis bone, skull, wrist, and other long bones. These digital images may also contribute to the identification of gender and age. In this paper, we have developed a system that makes the task easier in studying and analysing the femur digital radiographs for age and gender identification. This paper can be further carried out by developing a web-based application or on a smartphone-based application that can be user-friendly to access.

## Figures and Tables

**Figure 1:** FDI nomenclature illustrated on a panoramic radiograph.

**Figure 2:** Anatomy of human teeth.

**Figure 3:** Types of dental imaging. (a) Bitewing X-ray. (b) Periapical X-ray. (c) Orthopantomogram X-ray.

**Figure 4:** (a) Central incisor teeth measurement. (b) Intercanine measurement.

**Figure 5:** (a) and (b) Dataset distribution based on gender and age group.

**Figure 6:** Methodology for gender and age assessment system using OPG of teeth.

**Figure 7:** Dataset collected from College of Dental Science, Davangere.

**Figure 8:** Dataset collected from Bapuji Dental College and Hospital, Davangere.

**Figure 9:** Result of preprocessing.

**Figure 10:** Detection of edge in teeth image using Canny edge detector.

**Figure 11:** Feature matrix of teeth dataset for gender.

**Figure 12:** Feature matrix of teeth dataset for age.

**Figure 13:** Gender accuracy of teeth dataset.

**Figure 14:** Comparison of different LIBSVM kernels with different hyperparameter values. (a) Polynomial kernel, highest accuracy = 85.41% (*d* = 3, *c* = 28, and *g* = 0.81032). (b) Linear kernel, accuracy = 89.58% (*c* = 256). (c) RBF kernel, accuracy = 95% (*c* = 16; *g* = 0.08245). (d) Sigmoid kernel, accuracy = 83.33% (*c* = 512; *g* = 0.31626)).

**Figure 15:** Comparison of different MSVM kernels with different hyperparameter values. (a) Polynomial kernel, highest accuracy = 75.41% (*d* = 4, *c* = 64, and *g* = 0.09164). (b) Linear kernel, accuracy = 81.25% (*c* = 200). (c) RBF kernel, accuracy = 97.91(*c* = 45 and *g* = 0.043216). (d) Sigmoid kernel, accuracy = 87.50 (*c* = 24 and *g* = 0.32077).

**Table 1:** Numbering system and names of teeth.

	Maxillary jaw (upper jaw)			Mandibular jaw (lower jaw)		
	Universal numbering	Palmer numbering system	Tooth name	Universal numbering	Palmer numbering system	Tooth name
Right	1	Up. Rt. 8	3rd molar	32	L. Rt. 1	3rd molar
	2	Up. Rt. 7	2nd molar	31	L. Rt. 2	2nd molar
	3	Up. Rt. 6	1st molar	30	L. Rt. 3	1st molar
	4	Up. Rt. 5	2nd premolar	29	L. Rt. 4	2nd premolar
	5	Up. Rt. 4	1st premolar	28	L. Rt. 5	1st premolar
	6	Up. Rt. 3	Canine	27	L. Rt. 6	Canine
	7	Up. Rt. 2	Lateral incisor	26	L. Rt. 7	Lateral incisor
	8	Up. Rt. 1	Central incisor	25	L. Rt. 8	Central incisor
Left	9	Up. Lt. 1	Central incisor	24	L. Lt. 8	Central incisor
	10	Up. Lt. 2	Lateral incisor	23	L. Lt. 7	Lateral incisor
	11	Up. Lt. 3	Canine	22	L. Lt. 6	Canine
	12	Up. Lt. 4	1st premolar	21	L. Lt. 5	1st premolar
	13	Up. Lt. 5	2nd premolar	20	L. Lt. 4	2nd premolar
	14	Up. Lt. 6	1st molar	19	L. Lt. 3	1st molar
	15	Up. Lt. 7	2nd molar	18	L. Lt. 2	2nd molar
	16	Up. Lt. 8	3rd molar	17	L. Lt. 1	3rd molar

**Table 2:** Literature review summary.

SN	Authors	Year	Research findings	Remark
01	Saloni, Pradhuman V, P Mahajan, Ankush, Sukhleen Kaur, and Sakshi [16]	2020	Three parameters out of five mandible ramus variables studied showed statistically (*p* < 0.05) significant differences in gender	Mandible ramus may be used as an alternate tool in determining gender based on OPG
02	Poornima V, Surekha, Venkateswara Rao, G. Deepthi, Naveen S, and Arun Kumar [17]	2020	Right and left permanent mandible teeth were evaluated in OPG using the Camerier technique	High accuracy is achieved based on the Camerier method applied from an Indian-specific formula
03	A Okkesim and S Erhamza [18]	2020	The average value in min ramus width for males is 31.7 mm and for females is 29 mm. The average projection height value of ramus in females is measured 53.9 mm and in males is 48 mm	Mandible ramus in CBCT-based model exhibits significant differences in gender determination
04	N Vila, R. R. Vilas, and M. J. Carreira [19]	2020	Gender is evaluated based on DASNet and VVG 16 architecture	Accuracy of gender classification is 83% for DASNet and 90% for VGG-16
05	Vathsala Patil, Ravindranath, Saumya, Adithya, and Namesh [20]	2020	Gender determination based on mandible parameters using a logistic regression technique	In discriminant analysis, accuracy is 69%, in logistic regression, accuracy is 70%, and ANN shows the highest accuracy of 75%
06	J Albernaz, Nathalie A, Ferreira, Vanessa, and Proença [21]	2020	Teeth cast was used for the experimental procedure. Mesiodistal width of Rt. 1st molar to Lt. 1st molar was measured on each cast	Gender determination was classified with accuracy of 75%
07	Dalessandri D, Ingrid Tonni, Laura L, Marco Migliorati, Gaetano I, LVisconti, Stefano B, and C Paganelli [22]	2020	Reliability and accuracy of OPG versus CBCT for determination of age and gender	CBCT was found to be accurate when compared with OPG images in prediction
08	Stella A and Thirumalai [23]	2020	Tooth was divided into different stages starting from A stage to H stage	Individual age assessment using the Demirjian and the Nolla methods
09	Ahima Bali Behl [24]	2020	Measurement of bicondylar breadth (BB), gonial angle measurement, antegonial angle (AGA), ramus height, and ramus breadth (RHRB)	Upper and lower breadths of ramus were calculated. Ramus condylar height and coronoid height were measured appropriately
10	Vanessa M A, Rocharles, Andreia D'Souza, Casimiro, Andrea, Francisco C, and Deborah Q Eduardo Jr. [25]	2019	Equations for prediction of age and gender using pulp volumes from upper canine and upper central incisor	High accuracy can be achieved by using this formula when it is applied to pulp volume
11	Wallraff Sarah, Vesal Sulaiman, Syben Christopher, Lutz Rainer, and Maier Andreas [15]	2021	Unisex and sex-specific approaches based on deep learning methods achieve better results on the test data set	Male gender is slightly estimated younger than female gender

**Table 3:** Central incisor and intercanine width (male versus female).

Sl. no.	Parameters	Gender	Mean (in mm)
01	Central incisor width	Male	9.4
		Female	8.3
02	Intercanine distance	Male	29.14
		Female	25.7

**Table 4:** Class label description.

Class label	Gender
Class 0	Male
Class 1	Female

**Table 5:** MSVM class label description.

Class label_M	Age_M (years)	Class label_F	Age_G (years)
Class 1	1–15	Class 11	1–15
Class 2	16–20	Class 12	16–20
Class 3	21–25	Class 13	21–25
Class 4	26–30	Class 14	26–30
Class 5	31–35	Class 15	31–35
Class 6	36–40	Class 16	36–40
Class 7	41–45	Class 17	41–45
Class 8	46–50	Class 18	46–50
Class 9	51–55	Class 19	51–55
Class 10	56+	Class 20	56+

**Table 6:** LIBSVM testing for Gender with different kernels.

Kernel with hyperparameters	Number of samples correctly classified	Number of samples misclassified	Accuracy (%)
Linear (*C* = 256)	43	05	89.5833
Polynomial (*d* = 2, *C* = 64, *g* = 0.09153)	42	06	85.41
RBF (*C* = 16, *g* = 0.08245)	46	02	95.8333
Sigmoid (*C* = 512, *g* = 0.31626)	40	08	83.3333

**Table 7:** MSVM testing for age with different kernels.

Kernel with hyperparameters	Number of samples correctly classified	Number of samples misclassified	Accuracy (%)
Linear (*C* = 200)	39	09	81.25
Polynomial (*d* = 4, *C* = 64, and *g* = 0.05273)	36	12	75.0
RBF (*C* = 45 and *g* = 0.04317)	47	48	97.916
Sigmoid (*C* = 256 and *g* = 0.63419)	42	06	87.50

## Data Availability

The data that support the findings of this study are available from the corresponding author upon request.
